The article "Reconfigurable Architectures with High-Frequency Noise Suppression for Wearable ECG Devices" was published in 2021. Journal: J Healthc Eng.

# Reconfigurable Architectures with High-Frequency Noise Suppression for Wearable ECG Devices

**DOI:** 10.1155/2021/1552641

**Published:** 2021-12-22

**Authors:** V. Joseph Michael Jerard, M. Thilagaraj, K. Pandiaraj, M. Easwaran, Petchinathan Govindan, V. Elamaran

**Affiliations:** ^1^Department of ISE, Mangalore Institute of Technology and Engineering, Moodbidri, India; ^2^Karpagam College of Engineering, Coimbatore, India; ^3^Kalasalingam Academy of Research of Education, Srivilliputhur, India; ^4^Department of ECE, School of EEE, SASTRA Deemed University, Thanjavur, India; ^5^Department of Electrical and Electronics Technology, Ethiopian Technical University, Addis Ababa, Ethiopia

## Abstract

Recent advances in electronics and microelectronics have aided the development of low-cost devices that are widely used as well-being or preventive monitoring devices by many people. Remote health monitoring, which includes wearable sensors, actuators, and modern communication and information systems, offers effective programs that allow people to live peacefully in their own homes while also being protected in some way. High-frequency noise, power-line interface, and baseline drift are prevalent during the data-acquisition system of an ECG signal, and they can limit signal understanding. They (noises) must be isolated in order to provide an appropriate diagnostic of the patient. When removing high-frequency components (noise) from an ECG signal with an FIR filter, the critical path delay increases considerably as the filter's duration increases. To reduce high-frequency noise, simple moving average filters with pipelining and look-ahead transformation techniques are extensively used in this study. With the use of pipelining and look-ahead techniques, the only objective is to increase the clock speed of the designs. The moving average filters (conventional and proposed) were created on an Altera Cyclone IV FPGA EP4CE115F29C7 chip using the Quartus II software v13.1 tool. Finally, performance metrics such logic elements, clock speed, and power consumption were compared and studied thoroughly. The recursive pipelined 8-tap MA filter with look-ahead approach outperforms the other designs (685.48 MHz) in this investigation.

## 1. Introduction

Physiological factors are crucial indications of one's health. Electronic gadgets have long been used by doctors to aid in medical diagnosis by monitoring patients' biosignals and other bodily data. Issues such as global population aging, the frequency of chronic diseases, and the rapid expansion in healthcare needs have made remote patient surveillance a must to ensure that everyone receives high-quality care. As a result, there is a growing interest in home-based medical equipment that is both portable and reliable [1].

In the latest days, advances in wireless communication protocols have allowed these technologies to be integrated into a broad variety of medical devices. The data is delivered through communications infrastructure to monitoring locations, where a medical specialist or an intelligent system takes or processes the data acquired from various sensors or systems installed on/inside patients. Based on the application, the physician-patient contact will be developed immediately or soon using this data. Some of these techniques include cardiac hemodynamic monitoring. Some cardiac parameters, such as right ventricular pressure, right ventricle preejection time, and systolic time interval, are sensed in/on the body of individuals, such as the heart, arteries, and veins, and relayed to a monitoring station via wireless systems [2, 3].

Because of the requirement for regular inspection, their connection to hospital communication standards, and the usage of mobile phones and PDAs as clinical data terminals, personal sensor networks are becoming more widely used in clinical applications. Tiny size, power efficiency, lightweight, and interoperability with various mobile devices and communication networks are all requirements for a wearable device. The ability to perform real-time signal processing is also a significant aspect. Mobile communication has been increasingly popular in recent years. It can be a crucial component of the healthcare infrastructure. Heart diseases are on the rise as a result of industrialization. The difficulty of transportation, as well as the scarcity of cardiologists in several areas, has increased the demand for telehealth and computerized ECG analysis [4]. Few applications in wearable technology healthcare are shown in Figure 1.

Multiple aspects of the information technology profession and allied industry are being affected by technological advancements. The industry is currently being driven by performance level enhancement, computational time savings, ease of production, and end product portability. Wireless physiological signal monitoring is becoming more popular in personal medicine and home-based e-health systems [5]. The importance of physical well-being throughout treatment is becoming increasingly apparent. As a result, home care services are becoming increasingly popular. These technologies are designed to make it easier for doctors to keep track of their patients. The most critical information that doctors require is observed at the patient's home and transmitted to his doctor via the Internet. The main goal of this approach is to improve the person's health well-being by shortening his hospital stay. This might cut his treatment time in half [6, 7].

Many efforts have been made on biomedical projects today due to the medical complication and advancement in the field of medicine. It can provide the ideal environment for students who want to conduct cutting-edge research. Because of advances in medical image processing and its combination with modern technologies such as cloud computing, the medical industry has reached its pinnacle [8].  Figure 2 pinpoints a few applications of signal and image processing in the medical engineering field.

Signal and image processing is currently the most rapidly evolving domain in academia, research, and industry. In today's world of the medical engineering field, the analysis and processing of biosignals (pictures), as well as their clinical assessment (diagnosis), are critical. Since the advancement of computer technology, a plethora of tools have been made available for novices to investigate, study, and leverage any discipline of science and engineering [9, 10]. Digital signal processing (DSP) is a fast-evolving paradigm of estimation and filtering algorithms that are broadly employed in signal analysis and processing. Wireless communication systems design, advanced radar (sonar) systems, audio and speech signal processing, vibrations, imaging, biomedicine, and nondestructive control are just a few of the fields where DSP is often used [11, 12].

Different methods such as digital signal processing and image processing, wavelet transform, empirical mode decomposition, neural networks, and Markov models would help clinicians to secure a better clinical diagnosis. Rapid advancements in computational biology, biomechanics, biomedical, biological, diagnostic imaging, and numerical techniques have created a unique opportunity to leverage traditional computer models for a variety of biological systems to build modern diagnostic tools [13].

Because of the rise of artificial intelligence automation, biomedical engineering and technology are currently undergoing significant changes. Many obstacles in the field of biomedicine are being overcome thanks to modern machines and deep learning techniques. Biomedical engineering strikes a balance between engineering and medicine by combining engineering design and problem-solving methodologies with biological sciences to continue medical care, such as diagnosis, monitoring, and therapy [14]. Automated diagnosis approaches for a variety of medical problems would aid in the improvement of patient care. Biomedical data is frequently confronted with challenges such as the lack of elegant large database sizes, high-dimensional data, and class imbalance, to name a few [15]. In the fields of signals and systems, signal and image processing, digital signal processing, biomedical signal processing and control, and so on, simulation-based objects are widely applied.

Electronic health (E-health) and mobile health (M-health) have become more important in healthcare/telemedicine management systems, allowing clinicians and patients to research at their fingertips. In E-health applications, the advancement of wireless technology, notably smart devices, is critical [16]. New concepts such as “wireless hospital,” “mobile healthcare,” and “wearable remote monitoring” necessitate the creation of biosignal acquisition devices that can be successfully incorporated into medical practice [17].

The electrocardiogram (ECG) is a vital biological signal that is frequently utilized to make clinical diagnoses of cardiac conditions. Traditional ECG recorders send ECG data via wires, making them impractical for real-time monitoring in mobile scenarios or twenty-four-hour healthcare [18]. In recent years, wireless home care services have been widely discussed and are of interest in scientific and corporate researches. Wireless ECG recorders, like other wireless mobile systems, require power conservation for long-term use. As a result [19], a data compression technique can be utilized to save transmission energy while simply providing the RF module to communicate the most data with restricted bandwidth.

### 1.1. Related Previous Works

In this study [20], an ECG denoising method is presented. Their approach delivers great accuracy in the denoising of ECG data while consuming minimal CPU resources. Because the ECG signal contains high-frequency noise, often known as power-line interference, it must be eliminated before further processing can begin. This work describes a moving average filter-based technique for denoising high-frequency noise from an ECG signal. Following the filtering step, a polynomial curve fitting approach is used to smooth the ECG data.

Electrocardiogram (ECG) monitoring using portable equipment is complicated by motion artifacts, which can overlap the distinctive ECG waveforms. An adaptive filtering strategy for artifact removal is examined in [21] this paper. The method used makes use of motion-related data from an accelerometer linked to the ECG electrode. The experimental results show that using adaptive filtering to remove motion artifacts reduces the number of beat recognition errors, making our method an effective preprocessing scheme for ECG analysis. The created system, which was built on a commercial microcontroller, validated real-time requirements, resulting in a device that is suitable for portable monitoring [22].

The harder component of the filter design is that many real-time applications require the input data to be processed quickly. When using an FIR filter to remove high-frequency components (noise) from an ECG signal, the critical path delay grows dramatically as the filter's duration increases. In contrast to ordinary moving average filters, this study proved how to suppress noise using exponential averager approaches [23].

Power-line interference, baseline wandering, electromyogram noises, motion artifacts, and channel noises are some of the disturbances that can be contained in an ECG signal during acquisition and transmission. As a result, noise-free ECG readings are required for appropriate heart diagnosis. The main goal of this [22] study is to denoise the ECG signal, and the approach employed for this is empirical mode decomposition (EMD), which is ideal for any nonstationary signal because of its adaptive and data-driven character. Electromyogram noises (MA), motion artifacts (EM), and White Gaussian noises are among the high-frequency noises that have been studied for elimination. When the new algorithm is compared to current methods, encouraging results are produced, indicating that the proposed method is valid.

Due to the rapid growth of automation and artificial intelligence, biomedical engineering and technology are currently undergoing significant changes. While physiological recordings are made, the results are frequently contaminated by background noise or intrinsic interference in the recordings. The power-line interface and baseline wandering noise are common in electrocardiogram (ECG) data and can reduce the signal's intelligence. Although it is not possible to misinterpret the essential details more than indicated in standard guidance, the primary goal of this study is to use various filtering algorithms to reduce unwanted noise (baseline wandering). To eliminate the baseline wandering effect from an ECG signal, a DC bias elimination filter with various design structures [23] such as conventional, pipelined, look-ahead, and clustered look-ahead is used (clock speed).

The use of the first derivative of the filtered ECG with or without a moving average filter is advised for the QRS enhancement phase, but this approach [24] is vulnerable to noise and arrhythmia, necessitating the use of adaptive thresholding or integration-based approach for the detection phase. Both of the proposed approaches for detecting QRS complexes in mobile phone applications are simple and computationally efficient. Implementation of the original Pan-Tompkins method [25] is also a viable option if greater processing power is available, as it is on modern tablet computers and smartphones. Overall, building QRS detection algorithms for processing long-term recordings and big databases, as well as enhancing our telemedicine capabilities in the near future, requires simplicity and speed.

This article is organized as follows. The materials and methods are detailed in Section 2, which consists of the practical digital filtering experiments such as high-frequency noise removal from an ECG signal using simple moving average filters with various techniques. Simulation results and discussion with different performance measures are detailed in Section 3. Finally, the conclusions and future work are added in Section 4.

## 2. Materials and Methods

### 2.1. Framework of the Wireless Biosignal (ECG) Processing System

Rapid innovations in wireless communications and integrated circuits can enhance healthcare costs and management. The use of smart wearable electrocardiogram (ECG) equipment, for instance, can considerably improve the welfare of patients with cardiovascular disorders. Although enormous work has gone into the creation of such wearable devices, their incorporation into medical care is still limited, owing to difficulties of dependability and feasibility [26, 27].

Because of advancements in compactness and convenience, wearable sensors are becoming more common in health surveillance and human-machine interface technologies [28]. Latest innovations in flexible electronics have allowed the creation of wearable sensors that can dynamically bend and adapt to nonplanar and dynamic surfaces of the patient's psyche, enabling the measurement of physiological data with low bandwidth. Integrated systems have also been created, which combine movable sensors with inflexible computational components on a distinct substrate. These systems are ideal for applications requiring local signal processing and small form factors [29].

To create reliable and viable wearable ECG equipment, certain factors (in terms of power consumption, physical size, and cost) must be considered. Decreased power consumption, for example, would provide a longer battery life. The device's weight, dimensions, and affordability are all affected by its computational overhead. A wearable ECG device, as shown in Figure 3, is made up of numerous components in addition to the ECG electrodes (such as an analog interface and signal conditioning, and an A/D converter). The power usage, size, and expense of the device would all be affected by the hardware complexity of each of these building parts. The filtering block is one of the most important parts of wearable ECG equipment. Various types of noise and artifacts contaminate ECG signals, which must be eliminated and/or subdued using hardware efficient filters [30].

### 2.2. Related Works

The most common noninvasive diagnostic tool for identifying numerous cardiac illnesses is an electrocardiogram (ECG), which is a record of the heart's electrical activity over a while. It is a crucial component of a common e-health system, as ECG signals must frequently be compacted for lengthy data storage and distant delivery. High-speed parallel computes units, especially the field-programmable gate array (FPGA), and flexible software features are available with reconfigurable architecture [31, 32].

The FPGA is a reconfigurable computing device that is simply an integrated circuit (IC) that can be modified for any task. It is commonly used for prototyping and functional verification of ASICs (application-specific integrated circuits). FPGAs are significantly faster in applications where simultaneous computing is required for various processes due to their unique parallel computing capability [13, 33].

An e-health system is considered an integrated application of information technology and electronic communication in the health sector. It is a technology platform made up of diagnostic tools and microcomputers. e-health is a particularly important resource for persons in distant areas and impoverished countries, as it allows patients to consult with specialists via telecommunications. Electronic medical records are retained even in industrialized nations for follow-up therapy. As a result, the main system components of an e-health network are electronic communication and data recording [34].

ECG signals must be delivered to a remote site for telediagnosis and stored for future therapeutic reference as part of an e-health system. As a result, ECG signal reduction and a low-power acquisition method become necessary. Compression reduces the amount of bandwidth necessary for wireless communication, while low-power wireless technology helps to save money. It also reduces the amount of space required to store ECG data [35–37].

In the diagnosis of heart disorders, the electrocardiogram (ECG) is crucial. Cardiac illness and disorders are among the major causes of death around the world. Implantable and wearable ECG devices are becoming prominent instruments in real-time continuous disease diagnosis. Various sounds and artifacts, such as high-frequency noise, 60 Hz hum noise, baseline wandering, and radio frequency interference, commonly disrupt ECG signals during data acquisition. Significant characteristics of ECG signals are altered by these artifacts (noises). As a result, physicians seek noise-free ECG readings for effective diagnosis. As a result, multidisciplinary areas such as ECG signal processing are becoming more prominent in the physiological instrumentation industry and are receiving more special attention. Energy consumption, limited device size, speed, and price become significant challenges that must be carefully examined for such a critical (implantable ECG) usage.

EMD (empirical mode decomposition) is a relatively new algorithm. The EMD approach is fully based on data decomposition and is useful for nonstationary and nonlinear analysis [38, 39]. The EMD approach is also used to improve signal quality by reducing noise [40, 41]. Noises such as baseline drift and high-frequency components were removed from an ECG signal using an EMD-based method [42]. To remove noise from an ECG signal, some researchers used empirical mode decomposition and a moving average filter [43]; here, the existing EMD-based noise reduction was improved to improve performance. The EMD algorithms' primary flaw is the mode-mixing effect.

In recent years, there has been a significant increase in demand for digital signal processing optimized solutions, particularly in the fields of communication and current signal processing circuits. In the design of any sophisticated signal processing system, the finite impulse response (FIR) and infinite impulse response (IIR) filters are essential. The conventional moving average (MA) FIR filters, fast MA FIR filters using look-ahead arithmetic, conventional IIR filters utilizing a combination of integrator and comb sections (CIC) approach, and fast IIR filters using look-ahead arithmetic are all discussed in depth in this [44] work. These filters were created using an Altera EP4CE115F29C7 field-programmable gate array (FPGA) device and the Quartus II 13.1 synthesis tool. The conventional and fast MA FIR and IIR filters are compared in terms of performance measures such as the number of logic elements (LEs), performance, and power dissipation.

Pipelining IIR filters, on the other hand, is more complex and certainly not free. Simply adding pipeline registers to all adders will very certainly modify the pole locations and, as a result, the IIR filter's transfer function, especially in the feedback path. However, there have been reports in the literature of techniques that do not affect the transfer function while still allowing for better throughput. The following strategies have been described as promising for increasing IIR filter throughput [11]:

- Time-domain look-ahead interleaving
- Clustered look-ahead pipelining
- IIR decimation filter design
- Parallel processing
- Residue number system (RNS) implementation

Figure 4 depicts a typical ECG wave. The following are some key aspects of a typical clinical ECG:

- The peak voltage is usually around 1 mV
- The recommended sampling rate is 500 Hz
- Filtered bandwidth is around 0.05–100 Hz (for clinical)
- Filtered bandwidth is roughly 0.05–500 Hz (for high resolution)

Because the ECG signal contains high-frequency noise, also known as power-line interference, it must be filtered out for further processing during data collecting (better diagnosis). A simple moving average filter (low-pass filter) is employed to remove the high-frequency noise. Because of their huge benefits, such as linear phase reaction, assured stability, easier implementation, and reduced sensitivity to finite word-length problems, moving average (MA) filters are considered in this study.  Figure 5 shows the significant role of the MA filter for the removal of high-frequency contamination from an ECG signal.

In the literature, several approaches for reducing ECG signal noise have been investigated. For the reduction of noise in an ECG signal, few suggested an adaptive filtering method based on the discrete wavelet transform (DWT) and artificial neural networks (ANNs) [45]. The output signal-to-noise ratio was used to gain a large degree of signal amplification. Others introduced a noise reduction approach based on empirical mode decomposition (EMD) and discrete wavelet transform (DWT), which could recover all QRS complex wave properties from noisy ECG data [46].

When averaging, all data points have equal weight in a moving average, but, in a weighted moving average, the most recent (oldest) data point has the most higher (lower) weight. Exponential averaging is a type of average that reduces the delay caused by the moving average by giving the current data point a higher weight [47].

### 2.3. Proposed Low-Power Wireless Biosignal (ECG) Acquisition System

FIR (filters with a finite duration impulse response) and IIR (filters with an infinite duration impulse response) are the two types of digital filters. The existence of feedback in the IIR filter is the main distinction between the two filters. These two types of filters are fundamentally different, necessitating the employment of wholly separate design methodologies. The major focus of this paper is to construct and test an efficient 8-tap moving average (MA) filter on an FPGA device. The MA filters are the kind of finite impulse response (FIR).

#### 2.3.1. The Pipelined 8-Tap Moving Average Filter

Here, the pipelining technique is incorporated into the conventional 8-tap MA filter. The fundamental goal of implementing a pipelined system is to boost throughput.  Figure 6 shows the pipelined 8-tap MA filter.  Figure 7 depicts the RTL schematic view. The pipelined design achieves superior performance than the standard filter for obvious reasons. Various structures could, of course, be utilized in this case.

#### 2.3.2. The Pipelined 8-Tap Recursive MA Filter

Moving average filters are FIR filters, which are not recursive. FIR filters can also be implemented in a recursive style to save time on computation. The N-point MA filter, for instance, can be represented and shortened as [23, 48]

(1) $$\begin{array}{c} H\left(z\right)=\frac{1+z^{-1}+z^{-2}+z^{-3}+\cdots +z^{-\left(N-1\right)}}{N}\\ =\frac{1}{N}\sum_{n=0}^{N-1}{\left(z^{-1}\right)}^{n}\\ =\frac{1}{N}\left[\frac{1-z^{-N}}{1-z^{-1}}\right]. \end{array}$$

Similarly, a recursive form of an 8-tap moving average filter is as follows:

(2) $$\begin{array}{c} H\left(z\right)=\frac{1}{8}\left[\frac{1-z^{-8}}{1-z^{-1}}\right]. \end{array}$$

The (1–*z*^−8^) section acts as a comb filter, while the component 1/1 − *z*^−1^ acts as an integrator in this case. Cascade integrator comb (CIC) is the name given to this type of recursive moving average filter. The utility of an infinite impulse response (IIR) filter is also incorporated in the recursive kind of MA filter. That is, the FIR (comb) and IIR (integrator) parts are both present in the recursion. As a result, the pipelining may be readily applied to the FIR section, as can be seen in Figure 8.

#### 2.3.3. Look-Ahead Method on Pipelined Recursive MA Filter

The pipelining registers can be plugged into the FIR filter right away. However, to implement the pipelining notion in an IIR filter, another technique such as look-ahead transformation is required. As a result, the IIR portion of the recursive MA filter, as explained below, must be applied to this look-ahead transformation. In the time domain, the integrator portion (1/*z* − 1) is given as [23, 33]

(3) $$\begin{array}{c} y\left(n\right)=x\left(n\right)+y\left(n-1\right),\\ \text{or}\\ y\left(n+1\right)=x\left(n+1\right)+y\left(n\right). \end{array}$$

This can be stated as, using look-ahead transformation,

(4) $$\begin{array}{c} y\left(n+2\right)=x\left(n+2\right)+y\left(n+1\right). \end{array}$$

Using Equation (3)

(5) $$\begin{array}{c} y\left(n+2\right)=x\left(n+2\right)+x\left(n+1\right)+y\left(n\right). \end{array}$$

As a result, the output is

(6) $$\begin{array}{c} y\left(n\right)=x\left(n\right)+x\left(n-1\right)+y\left(n-2\right). \end{array}$$

The recursive moving average filter (8-tap) with CIC style and look-ahead transformation is shown in Figure 9.

## 3. Results and Discussion

The principal goal of this research is to construct and test an affordable 8-tap moving average (MA) filter on an Altera FPGA device. The functionality of the MA filters was assessed using a very high-speed integrated circuits hardware description language (VHDL) on an Altera DE2–115 FPGA (EP4CE115F29C7) device for FPGA implementation (VHDL).  Figure 10 shows the Altera DE2-115 FPGA board which is used in this study [49]. The following are the primary needs for a real-time filter [50]:

- Smaller area
- Less energy use
- Lower delay (higher performance)

### 3.1. Performance Measures

For assessing (comparing) experimental results among the filters, the following three performance metrics were used [51, 52].

#### 3.1.1. Logic Elements

Prefabricated logic blocks, connection resources, and input/output (IO) blocks are all common features of FPGAs. The utilization report for resources (LEs), which can be triggered by synthesis tools, would aid in determining the number of logic elements required for the design.

#### 3.1.2. Critical Path Delay

The path with the longest delay is referred to as a crucial path in the design. Computing the reciprocal of the critical path delay determines the design's performance or speed. For example, if the critical path delay is estimated to be 2.65 ns, the performance will be 377.35 MHz.

A further important implication on critical path delay is illustrated in Figure 11. There is a longer critical path delay (14.381 ns) and worse performance as a result of adding first and then dividing. Hence, the performance becomes the reciprocal of 14.381 ns (69.53 MHz).

#### 3.1.3. Registers

A register is a collection of flip-flops that keeps track of a bit pattern. A clock, input data, output data, and enable signal port are all included in a register on the FPGA. The input data is latched and saved inside every clock cycle, and the output data is updated to reflect the internally stored data [53].

#### 3.1.4. Power Dissipation

With the FPGA platform, power consumption is also a major design constraint. Static and dynamic powers are the two types of power available. The first is independent of the design; in other words, even unused logic blocks would be using static power. The second is entirely design-dependent; i.e., it varies depending on clock frequency, device utilization, and other resources such as RAM, PLL, and embedded multipliers. In addition, the I/O (input/output) power appears as a result of the design's number of I/O pins.

### 3.2. The Pipelined 8-Tap MA Filter

The fundamental goal of implementing a pipelined system is to boost throughput.  Table 1 shows a considerable difference in clock speed (highlighted in bold) between the pipelined and conventional designs, indicating that the pipelined design outperforms the conventional design. In other words, when compared to the nonpipelined design, the pipelined architecture achieves a speed-up of around 142 percent. For obvious reasons, the logic elements (156) and the registers (119) in the pipelined approach are slightly higher than the conventional design. The total power dissipation, which includes dynamic power, static power, and I/O power, becomes 137.74 mW for the pipelined approach [48].

### 3.3. The Pipelined 8-Tap Recursive MA Filter

Further to improve the performance, the pipelining concept is incorporated an 8-tap recursive MA filter. The simulation results on both are compared in Table 2. It shows a significant difference in performance (highlighted in bold) between the pipelined and conventional designs, representing the fact that the pipelined design obtains better performance than the conventional design [54]. That is, when compared to the nonpipelined design, the pipelined architecture produces a speed-up of around 89 percent. As seen in Table 2, as the complexity of the problem grows, so does the requirement for memory bits. The total power dissipation, which includes dynamic power, static power, and I/O power, becomes 138.67 mW for the pipelined approach.

### 3.4. The Pipelined Recursive MA Filter with Look-Ahead Approach

Further to enhance the performance, the look-ahead technique concept is embedded into an 8-tap pipelined recursive MA filter. The simulation results on both are summarized in Table 3. It shows a slight improvement in the clock speed (highlighted in bold) between the look-ahead and conventional designs, representing the fact that the proposed method obtains higher performance than the conventional one. In other words, when compared to the conventional design, the look-ahead approach produces a speed-up of around 6.7 percent. As seen in Table 3, the number of memory bits required increases as the problem becomes more difficult. The total power dissipation, which includes dynamic power, static power, and I/O power, becomes 138.81 mW for the look-ahead approach. The pipelined recursive MA filter with a proposed approach obtains higher performance results at the cost of more logic elements (83) and registers (78), as expected. This study, too, has significant limitations for various reasons. In the case of moving average FIR filters, for instance, the parallel and transposed structures were not investigated. There are so many significant comparisons among the power dissipation data because the filters were deployed in an FPGA device. Instead, the filters can be used in application-specific integrated circuits (ASIC) for better outcomes (space, speed, and power).

### 3.5. Limitations

This study, too, has significant limitations for obvious reasons. In the case of moving average FIR filters, for example, the parallel and transposed structures were not investigated. There are so many significant comparisons among the power dissipation data because the filters were deployed in an FPGA device [55]. Instead, the filters can be used in application-specific integrated circuits (ASIC) for better results (space, speed, and power).

## 4. Conclusion

The majority of real-time applications necessitate quick input data processing, which is the most difficult element of the filter design process. The critical path delay in an FIR filter, for example, grows dramatically as the filter length increases. To improve the performance of DSP circuits, popular high-speed techniques such as pipelining and look-ahead transformation are used (digital filters). In the future, powerful electronic computer automated design (ECAD) techniques could be used to implement the proposed filter architectures in ASIC style approaches. Also, this approach could be expanded to eliminate other disturbances such as power-line interference and EMG noise. This work can be expanded to other ideas in digital signal processing, such as the half-band filter, digital Hilbert-transform filter, multirate filter banks, least-mean-squares (LMS) filters, and Goertzel algorithm, using FPGA architecture. The major goal is to demonstrate the benefits of FIR filter design techniques, such as low-power consumption, lower area, and excellent performance. This research can be used to create fast digital infinite impulse response (IIR) filters, multirate signal processing, and filter banks, among other things.

## Figures and Tables

**Figure 1:** Wearable technology in healthcare.

**Figure 2:** Applications of signal and image processing in healthcare.

**Figure 3:** Wearable ECG devices transmit the collected data to a remote backend system for additional processing (through a cellular network).

**Figure 4:** A typical ECG wave.

**Figure 5:** The removal of high-frequency noise from an ECG. (a) Actual ECG signal. (b) Filtered ECG signal by the 8-tap moving average filter.

**Figure 6:** The pipelined 8-tap moving average filter.

**Figure 7:** RTL schematic view of a pipelined 8-tap moving average filter.

**Figure 8:** The pipelined recursive 8-tap MA filter using the CIC method.

**Figure 9:** The pipelined recursive 8-tap MA filter using CIC and look-ahead transformation.

**Figure 10:** Altera DE2-115 FPGA board.

**Figure 11:** More critical path delay by sum and divide approach.

**Table 1:** Simulation Results of an 8-tap MA filter (conventional vs. pipelined).

Measures	Conventional (without pipelining) [54]	With pipelining [48]
Logic elements	154	156
Registers	106	119
Power dissipation	135.57 mW	137.74 mW
Performance (clock speed)	87.71 MHz	**211.10 MHz**

**Table 2:** Simulation Results of a recursive 8-tap MA filter (conventional vs. pipelined).

Measures	Conventional (without pipelining)	With pipelining
Logic elements	68	66
Registers	48	48
Memory bits	75	90
Power dissipation	138.03 mW	138.67 mW
Performance (clock speed)	339.90 MHz	**642.67 MHz**

**Table 3:** Simulation Results of a recursive pipelined 8-tap MA filter (typical vs. look-ahead).

Measures	Conventional (without look-ahead)	With look-ahead
Logic elements	66	83
Registers	48	78
Memory bits	90	90
Power dissipation	138.67 mW	138.81 mW
Performance (clock speed)	642.67 MHz	**685.48 MHz**

## Data Availability

The data used to support the findings of this study are available from the corresponding author upon request.
